The article "Construction of College English Teaching Environment Assessment Model Based on BP Neural Network and Multiple Intelligence Theory" was retracted in 2023. Reasons: signs of a paper mill; suspected computer-generated content; unreliable results or conclusions; lack of ethics approval or compliance.

# Construction of College English Teaching Environment Assessment Model Based on BP Neural Network and Multiple Intelligence Theory

**DOI:** 10.1155/2022/9479755

**Published:** 2022-09-09

**Authors:** Hailong Li

**Affiliations:** Liaocheng University Dongchang College, Liaocheng 252000, China

## Abstract

College English has almost always been a required course, and a college student's level of English proficiency is one of the factors used to assess their learning capacity. The quality of students' English learning is largely influenced by the level of English instruction provided in colleges. However, there are still a lot of issues with college English instruction today, the most glaring of which is that English instruction is being overly simplified, and that the methods, modes, and purposes of instruction are also very narrow. Due to this, it is challenging for most colleges and universities' English teaching levels to satisfy the requirements of high-level education. The PSO-BP neural network model, which optimizes the BP neural network (BPNN), is used in this study to build a high-precision and diversified English teaching evaluation model in order to address the aforementioned issues. According to the experimental findings, the PSO-BPNN algorithm has a relative error of just 0.29 percent and an average accuracy rate of 97.02 percent. Overall performance is superior to that of the conventional BPNN algorithm, and it is the most adaptable in terms of creating various evaluation modes.

## 1. Introduction

In college English courses, the single teaching mode has been widely criticized as a defect. Simplification will cause English teaching to lose interest and attractiveness, and students' learning status will also be greatly affected. In the past, English teachers only focused on instilling knowledge in the classroom. Most of the time, they ignored the interaction with students and how to stimulate students' interest in learning. How to make teaching fun is often a difficult problem. In this case, it is necessary to construct a diversified English teaching model. It can enrich the teaching links and at the same time allow students to be well integrated into the whole teaching atmosphere, giving students a strong sense of participation, rather than only teachers leading the whole process. At the same time, in this mode, test scores are no longer the only assessment criteria. The diversified assessment system will give students more motivation to study and promote their all-round development. In view of the above problems, in order to improve the scientificity and accuracy, considering that the BP neural network can well improve the accuracy of the corresponding model and reduce the error, this paper proposes a BPNN related model to construct a multivariate evaluation model.

The article "Construction of College English Teaching Environment Assessment Model Based on BP Neural Network and Multiple Intelligence Theory" was retracted in 2023. Reasons: signs of a paper mill; suspected computer-generated content; unreliable results or conclusions; lack of ethics approval or compliance.

This paper constructs the teaching evaluation model in university English based on the BPNN correlation model. The purpose is to change the shortcomings of the previous college teaching in English that is too simplistic, to make diversified improvements to classroom teaching and student evaluation models, to stimulate students' learning motivation, and to promote the all-round development of students' English proficiency. The innovation of this paper is that (1) the theory of multiple intelligences is applied to the construction of the multiple evaluation models, which makes the whole model more theoretical basis. (2) Combined with the PSO algorithm, the original BP network model can be optimized, which can greatly improve the data accuracy and reduce the experimental error.

## 2. Related Work

Because college English is basically a compulsory course for every college student, the quality of English teaching affects students' class experience and knowledge absorption to a large extent. Therefore, in recent years, how to construct an excellent teaching evaluation model in university English has been deeply concerned and researched by relevant scholars. Among them, scholar Jinyu pointedly put forward the introduction of summative assessment theory in college teaching in English, and analyzed the feasibility of applying this method to college English classrooms. He constructed a teaching model in university English based on this theory and checked the validity of the model through relevant experiments [1]. Tran et al. conducted a related discussion on English teaching school. It mainly reviews the role of English school-based in English teaching and students' English learning, and analyzes the impact of school-based assessment strategies on teachers' decision-making. They finally discussed the relationship between school-based evaluation and English teaching evaluation model [2]. Nguyen creatively proposed to introduce an alternative evaluation method into the English teaching evaluation model through a questionnaire survey on English teaching innovation of English teachers in a public middle school, and discussed the feasibility of this method in depth [3]. Ernawati et al., aims at exploring new and feasible ways of evaluating multiple intelligences. By analyzing relevant literature and conducting professional interviews with relevant English teaching professionals, it can obtain an effective method for students' English teaching. This method can be used to identify students' intelligence, perception, and other related abilities [4]. Koroleva considered and analyzed an increasingly popular model of authentic foreign language teaching assessment–the formation of educational profiles. He provided and summarized examples of the practical application of this real-world foreign language teaching assessment model in teaching business English to students pursuing a bachelor's degree in tourism and English for specific purposes to students pursuing a master's degree in jewelry [5]. The above research on the evaluation model of teaching English at the University has enriched the relevant theoretical basis of the evaluation model of teaching to a great extent. It fully embodies the advantages of diversity and plasticity of teaching evaluation, and provides great help to the establishment of a multievaluation system for English teaching. However, the above studies do not combine the theory of multiple intelligences with the multiple evaluation system. This will lead to superficial research, and cannot create a truly comprehensive and diversified English teaching evaluation model, which will make English teaching too single. At the same time, the data accuracy of the evaluation model created by the above research is not high enough to reflect the scientific nature of the algorithm.

The article "Construction of College English Teaching Environment Assessment Model Based on BP Neural Network and Multiple Intelligence Theory" was retracted in 2023. Reasons: signs of a paper mill; suspected computer-generated content; unreliable results or conclusions; lack of ethics approval or compliance.

Aiming at the problem that the data accuracy mentioned above is difficult to achieve the expected, BPNN can be used to solve this problem. BPNN can improve the accuracy of experimental data and reduce the relative error, which is very suitable for studying similar projects with high data accuracy requirements. Therefore, many experts and scholars have conducted in-depth discussions on the knowledge of BPNN. Among them, scholar Lü et al. used LM-BPNN to fit the experimental results. They used the LM-BPNN to fit *S*-wave velocities under multiple conditions for higher accuracy, estimating an average relative error of 2.22% [6]. Zhang et al. optimized the weight and threshold selection process of the BP network to improve the inversion results. Then, a better network model is obtained, and the model is used for the inversion of the density interface model, which can improve the inversion accuracy [7]. Considering the complexity and variability of fire risk factors, Liu et al. proposed a forest fire risk assessment model based on BPNN for transmission lines. Combined with the actual situation of the fire, the actual situation of some 220 kV and above transmission lines in areas with high incidence of forest fires, several factors and the actual fire assessment level are selected as the input and output of the model [8]. Zeng et al. proposed an early warning control strategy based on BPNN optimized by genetic algorithm. They introduced the BPNN optimized by genetic algorithm to optimize the traditional TTR algorithm [9]. Scholar Hu et al. optimized and introduced a GA-BPNN model based on the original neural network, which can be used to test the noise situation of the motor, and creatively realize the prediction function. In comparison, the experimental results show that the maximum difference between the two is only less than 5 decibels [10]. The above research on BPNN provides strong data support and theoretical enrichment for the practical application of BPNN, and helps relevant researchers to better understand and use the BPNN architecture. The BP network architecture in the above-mentioned related research still has shortcomings such as slow convergence speed and easy to fall into the local minimum, which is still not enough to support the research on the related college English teaching multiassessment model.

The article "Construction of College English Teaching Environment Assessment Model Based on BP Neural Network and Multiple Intelligence Theory" was retracted in 2023. Reasons: signs of a paper mill; suspected computer-generated content; unreliable results or conclusions; lack of ethics approval or compliance.

## 3. Design and Construction of Multiassessment Model for College Teaching in English Based on BPNN

### 3.1. Construction of Multiple Evaluation Models for College Teaching in English

The emphasis of the education sector has always been on English college teaching. The effectiveness of English instruction has an impact on students' learning progress as well as the future planning and trajectory of their entire university careers. The way English is taught at the moment is far too basic; all that is involved is the old-fashioned method of lecturing and listening on the part of the teacher. This is very detrimental to students' learning in English classes and does not maximize their learning potential. Therefore, a challenging issue that needs to be resolved is how to create a thorough and varied English teaching evaluation model. This essay combines “multiple intelligences” theory to create a multiassessment system for college English teaching with the goal of offering an effective and workable solution to the aforementioned issues.

#### 3.1.1. Overview of Multiple Intelligences Theory

The theory of multiple intelligences has been proposed as early as the 20th century. It points out that the intelligence possessed by human beings is not only one but consists of eight or more intelligences, which are independent of each other and have no special dependence, as shown in Figure 1. This theory is put forward to show that people can solve problems encountered in life, work and other affairs through their own multiple intelligence abilities. As can be seen from Figure 1, the eight kinds of intelligence possessed by humans are all equally important, and the details are as follows:

1. linguistic intelligence: the ability to organize and express language clearly, including spoken and unspoken language.
2. Logical and mathematical intelligence: the ability to fully understand logical relationships, solve mathematical problems well, and understand the causal relationship of things.
3. Visual/spatial intelligence: give full play to visual performance, have good spatial construction and spatial analysis capabilities, fully understand spatial geometry, graphics, and visual knowledge, and have good construction capabilities for architecture, painting, and images.
4. Musical intelligence: the ability to have strong control over music, melody, rhythm, etc.
5. Physical kinesthetic intelligence: the ability to use the body flexibly, has strong physical coordination, and use the whole body to perceive things.
6. Naturalistic intelligence: have a strong perception of nature, be able to recognize the natural environment freely and be aware of nature.
7. Interpersonal intelligence: the ability to get along well with others, to handle interpersonal relationships well, and to make oneself popular.
8. Introspective intelligence: the ability to sense one's own feelings, reactions, and motivations in time, with strong self-awareness.

The article "Construction of College English Teaching Environment Assessment Model Based on BP Neural Network and Multiple Intelligence Theory" was retracted in 2023. Reasons: signs of a paper mill; suspected computer-generated content; unreliable results or conclusions; lack of ethics approval or compliance.

As can be seen from Figure 1, the eight kinds of intelligence possessed by humans are all equally important, and the details are as follows. Among these eight kinds of intelligence, linguistic intelligence, visual-spatial intelligence, musical intelligence, interpersonal intelligence, and introspection intelligence are all positively correlated with college teaching in English. Introducing the concept of multiple intelligences into the classroom teaching and teaching evaluation of foreign language in colleges and universities can help teachers deeply understand students' learning preferences and better appreciate their intellectual advantages. The purpose of teaching evaluation is to provide students with beneficial feedback through various evaluations, so that students can develop their intellectual advantages. It can stimulate their enthusiasm for learning and improve their learning efficiency, so as to truly achieve the purpose of promoting construction and learning through evaluation.

#### 3.1.2. Construction of a Multiassessment System for College Teaching in English

In order to avoid the situation of English teaching being too simple, this paper will start from three aspects: teaching mode, teaching method, and teaching purpose of English teaching. The purpose is to solve the three major drawbacks of English teaching that the previous teaching mode is mainly based on knowledge instillation, focusing on imparting knowledge, teaching methods relying on a single grammar translation method, and the teaching purpose is mainly selecting talents. The specific English teaching multimode is shown in Figure 2.

The article "Construction of College English Teaching Environment Assessment Model Based on BP Neural Network and Multiple Intelligence Theory" was retracted in 2023. Reasons: signs of a paper mill; suspected computer-generated content; unreliable results or conclusions; lack of ethics approval or compliance.

Figure 2 shows the English teaching multiassessment system constructed in this paper. From the three aspects of teaching mode, teaching purpose, and teaching method, it abandons the shortcomings of most college teaching in English which are monotonous and ineffective. Combined with the theory of multiple intelligences, the idea of using multiple intelligences in teaching is proposed in an original way, aiming at improving students' all-round abilities and promoting students' all-round development. In the end, each student's English learning ability and English use level will be improved. The following is a detailed introduction to the system.

The multiassessment system of college teaching in English proposed in this paper not only takes the students' final exam scores as the only evaluation standard but also incorporates other evaluation indicators to comprehensively consider the students' English learning level. It includes the usual classroom performance, teachers' comprehensive evaluation scores for students, mutual evaluation scores among students, and students' self-evaluation scores. In addition, a comprehensive assessment exam will be set up midterm. The content of the test not only includes the English reading, writing, listening, and speaking of the traditional test but also adds the assessment of the students' eight multiple intelligences. For students' performance of different multiple intelligences in English classrooms, for example, singing English songs shows students' musical intelligence, speaking fluently in English in class shows students' language intelligence, and cooperating with team members in English group cooperation shows students' interpersonal intelligence. Teachers and classmates can record and score students' multiple intelligences. The final assessment results are shown in Table 1.

As can be seen from Table 1, students' final exam scores are no longer the only criterion for evaluating a student's English learning level and ability. Although this indicator still accounts for the largest proportion of 50%, other indicators also play an important role in the final English score of students. This means that a student's final exam scores are high but others are mediocre, which does not mean that the student's English proficiency is high. In this evaluation mode, students' English scores are freed from the shackles of simplification. Instead, students' standards are evaluated in a diversified manner from the perspective of students' overall development. This is conducive to mobilizing students' enthusiasm, tapping their English learning potential, and helping students move towards a higher level of English learning platform.

The article "Construction of College English Teaching Environment Assessment Model Based on BP Neural Network and Multiple Intelligence Theory" was retracted in 2023. Reasons: signs of a paper mill; suspected computer-generated content; unreliable results or conclusions; lack of ethics approval or compliance.

### 3.2. Construction of BPNN

The basic model of BPNN consists of three parts [11, 12]. The first part is the input layer, which is used to accept valid information, and the second part is the hidden layer. It is used to process the received information, and the last one is the output layer that summarizes and outputs the processing results. Its basic structure is shown in Figure 3.

It can be seen from Figure 3 that the number of hidden layers is larger than that of the input layer and the output layer, and the nodes of the hidden layer are connected to the nodes of each input layer and output layer. In this way, a complete basic model of BPNN can be formed.

In the BPNN, the number of nodes in the input layer, hidden laye,r and output layer are set as *m*, *n*, and *k*, respectively. At the same time, set the connection weight between the input layer and the hidden layer connection node to *W*_ji_, also set the connection weight between the output layer and the hidden layer connection node to *φ*_*hj*_, and then calculate the output of the hidden layer node, which is represented by *v*_*j*_:

(1) $$\begin{array}{c} v_{j}=f_{a}\left(\overset{m}{\underset{i=0}{\sum }}W_{ji}y_{i}\right). \end{array}$$

In equation (1), the function *f*_*a*_ is used to represent the transfer function of the hidden layer [13], and the processing function used to process the data in the output layer is set to *f*_*b*_, and then the final output parameters are derived from the equation:

(2) $$\begin{array}{c} z_{h}=f_{b}\left(\overset{n}{\underset{j=0}{\sum }}\varphi_{hj}v_{j}\right). \end{array}$$

Introduce input learning samples [14], denoted by *Q*, convert *Q* into corresponding data through *y*^1^, *y*^2^, ⋯, *y*^*q*^, and then, use the data for BPNN to obtain the actual output value of *z*_*h*_^*q*^. Then, set the learning rate parameter *γ* to derive the expected output value *e*_*h*_^*q*^, and bring the *e*_*h*_^*q*^ sum of the obtained *z*_*h*_^*q*^ into the squared error equation together to obtain the final result of the *Q* sample:

(3) $$\begin{array}{c} F_{q}=\frac{1}{2}\overset{k}{\underset{h=1}{\sum }}{\left(e_{h}^{q}-z_{h}^{q}\right)}^{2}. \end{array}$$

In the *Q* sample, the global error [15] is formulated as:

(4) $$\begin{array}{c} F=\frac{1}{2}\overset{q}{\underset{q=1}{\sum }}\overset{k}{\underset{h=1}{\sum }}{\left(e_{h}^{q}-z_{h}^{q}\right)}^{2}=\overset{q}{\underset{q=1}{\sum }}F_{q}. \end{array}$$

The output layer weight *φ*_*hj*_ is adjusted according to the accumulated result of a single error calculated in the sample, in order to reduce the global error *F* and improve the sample accuracy [16]:

(5) $$\begin{array}{c} \Delta \varphi_{hj}=\overset{q}{\underset{q=1}{\sum }}\left(-\gamma \frac{\partial F}{\partial \varphi_{hj}}\right). \end{array}$$

Next, define the error signal as:

(6) $$\begin{array}{c} \chi_{zh}=-\frac{\partial F}{\partial T_{h}}. \end{array}$$

To derive equation (6), first,

(7) $$\begin{array}{c} \frac{\partial F_{q}}{\partial z_{h}}=-\overset{k}{\underset{j=1}{\sum }}\left(e_{h}^{q}-z_{h}^{q}\right). \end{array}$$

Then,

(8) $$\begin{array}{c} \frac{\partial z_{h}}{\partial T_{h}}=f_{b}\left(T_{h}\right). \end{array}$$

Equation (8) represents the outlier component of the correlation function used to transfer the effect in the output layer of the network [17], from which it can be obtained:

(9) $$\begin{array}{c} \chi_{zh}=\overset{k}{\underset{h=1}{\sum }}\left(e_{h}^{q}-z_{h}^{q}\right)f_{b}\left(T_{h}\right). \end{array}$$

Then, according to the chain theorem [18], we can get:

(10) $$\begin{array}{c} \frac{\partial F_{q}}{\partial \varphi_{hj}}=-\overset{k}{\underset{h=1}{\sum }}\left(e_{h}^{q}-z_{h}^{q}\right)f_{b}\left(T_{h}\right)v_{j}. \end{array}$$

According to equation (10), the weight change of the output layer is expressed as:

(11) $$\begin{array}{c} \Delta \varphi_{hj}=\overset{q}{\underset{q=1}{\sum }}\overset{k}{\underset{h=1}{\sum }}\gamma \left(e_{h}^{q}-z_{h}^{q}\right)f_{b}\left(T_{h}\right)v_{j}. \end{array}$$

Then, let Δ*W*_*ji*_ be expressed as the weight change of the hidden layer, as follows:

(12) $$\begin{array}{c} \Delta W_{ji}=\overset{q}{\underset{q=1}{\sum }}\left(-\gamma \frac{\partial F_{q}}{\partial W_{ji}}\right). \end{array}$$

The error signal is represented by *χ*_*vj*_:

(13) $$\begin{array}{c} \chi_{vj}=-\frac{\partial F_{q}}{\partial T_{j}}. \end{array}$$

Among them,

(14) $$\begin{array}{c} -\frac{\partial F_{q}}{\partial v_{j}}=-\overset{k}{\underset{h=1}{\sum }}\left(e_{h}^{q}-z_{h}^{q}\right)\frac{\partial z_{h}}{\partial z_{j}}. \end{array}$$

The chain theorem is a derivation rule used in the derivation of calculus. The chain theorem looks like this:

(15) $$\begin{array}{c} \begin{array}{c} \frac{\partial z_{h}}{\partial v_{j}}=f_{b}\left(T_{h}\right)\varphi_{hj},\\ \frac{\partial v_{h}}{\partial T_{j}}=f_{b}\left(T_{h}\right). \end{array} \end{array}$$

It is the partial differential representation of *f*_*a*_, therefore,

(16) $$\begin{array}{c} \chi_{vj}=-\frac{\partial F_{q}}{\partial T_{j}}=\overset{k}{\underset{h=1}{\sum }}\left(e_{h}^{q}-z_{h}^{q}\right)f_{b}\left(T_{h}\right)\varphi_{hj}f_{a}\left(T_{j}\right). \end{array}$$

Then, it can be deduced from the chain theorem:

(17) $$\begin{array}{c} \frac{\partial F_{q}}{\partial W_{ji}}=-\overset{k}{\underset{h=1}{\sum }}\left(e_{h}^{q}-z_{h}^{q}\right)f_{b}\left(T_{h}\right)\varphi_{hj}f_{a}\left(T_{j}\right)y_{i}. \end{array}$$

According to equation (17), Δ*W*_*ji*_ changes as follows:

(18) $$\begin{array}{c} \Delta W_{ji}=\overset{q}{\underset{q=1}{\sum }}\overset{k}{\underset{h=1}{\sum }}\left(e_{h}^{q}-z_{h}^{q}\right)f_{b}\left(T_{h}\right)\varphi_{hj}f_{a}\left(T_{j}\right)y_{i}. \end{array}$$

The BPNN can improve the accuracy of the multivariate evaluation mode, but when it falls into a local minimum deadlock, it cannot maintain the high accuracy. The reason is that the local deadlock will affect the selection of initial weights, and if the selected values are of different sizes, the local minima will also change.

The article "Construction of College English Teaching Environment Assessment Model Based on BP Neural Network and Multiple Intelligence Theory" was retracted in 2023. Reasons: signs of a paper mill; suspected computer-generated content; unreliable results or conclusions; lack of ethics approval or compliance.

### 3.3. Construction of PSO-BPNN

The previous section expounded that the BPNN is prone to the situation that the accuracy cannot meet the system requirements when the initial weights are indeterminate, and the final experiment may not reach the expected value of the multiassessment model for college teaching in English constructed in this paper. Therefore, this paper proposes a PSO-BPNN, as shown in Figure 4. It is an improved algorithm based on BPNN.

Figure 4 shows the structural composition of the PSO-BPNN. It adds feedback mechanism on the basis of BPNN and has adaptive learning ability. It can give feedback according to the results of the output layer and continuously adjust the weight of the corresponding parameters, so that the output vector and the expected vector can reach an ideal difference.

First, the equation planning of the three-layer architecture of the BPNN is carried out by the least square method [19]. Assuming that the particle swarm consists of *n* particles, then, *n* particles represent *n* corresponding feasible solutions. The *c*-dimensional position vector of the *i*th particle is represented by *v*_*i*_ = (*v*_*i*1_ + *v*_*i*2_, ⋯, *v*_*iC*_), the flying speed of the particle is represented by *s*_*i*_ = (*s*_*i*1_, *s*_*i*2_, ⋯, *s*_*iC*_), the best position of the particle can be represented by *p* − optimal_*i*_ = (*p*_*i*1_, *v*_*i*2_, ⋯, *p*_*ic*_, ⋯, *p*_*iC*_), and the best position expression of the entire particle group is *t* − optimal_*i*_ = (*t*_*i*1_, *t*_*i*2_, ⋯, *t*_*ic*_, ⋯, *t*_*iC*_).

The updated expression of the particle velocity is:

(19) $$\begin{array}{c} s_{ic}^{h+1}={RS}_{ic}^{h}+a_{1}u_{1}\left(p_{ic}-v_{ic}^{h}\right)+a_{2}u_{2}\left(t_{c}-v_{ic}^{h}\right). \end{array}$$

The updated expression for the particle position is:

(20) $$\begin{array}{c} v_{ic}^{h+1}=v_{ic}^{h}+s_{ic}^{h+1}. \end{array}$$

In equation (19), the iteration number is represented by *h*, and the inertia weight is represented by *R*. Two numbers are randomly selected in the interval [0, 1], set as *u*_1_ and *u*_2_, the learning factor is denoted as *a*_1_, and the acceleration coefficient is denoted as *a*_2_. Usually, the initial value is set to *a*_1_ = *a*_2_ = 1. The position of the particle in the total sample can be expressed as a set of BP weights and thresholds, and then an initial value is assigned to the example position, which can be established by scanning the weight matrix and threshold in the neural network [20–22].

(21) $$\begin{array}{c} s_{ic}^{h+1}=\varphi s_{ic}^{h}+a_{1}u_{1}\left(p_{ic}-v_{ic}^{h}\right)+a_{2}u_{2}\left(t_{c}-v_{ic}^{h}\right). \end{array}$$

The iteration is done according to equations (20) and (21):

(22) $$\begin{array}{c} \gamma =\gamma_{\max}-\frac{\gamma_{\max}-\gamma_{\min}}{h_{\max}}\times h. \end{array}$$

The weight of particle velocity iteration is represented by *γ*, equation (22) is the calculation equation of *γ*, and *γ*_max_ represents the weighted value. *γ*_min_ represents the final calculated weighted value, *h* represents the number of iterations that have been performed currently, and *h*_max_ represents the largest value among all iterations. In the research process, the BPNN model is combined with the PSO algorithm and the weights and thresholds of the model are trained, and finally, calculate the optimal position when all particles are optimized [23].

(23) $$\begin{array}{c} \varphi_{i,m}^{h+1}=\varphi_{i,m}^{h}+s_{ic}^{h+1}. \end{array}$$

Equation (23) represents the learning equation of weights and thresholds in the neural network, where the corresponding velocity of the particle in the *h* + 1-th iteration is represented by *φ*_*i*,*m*_^*h*^, and the corresponding weight of the particle in the *h*-th iteration is represented by *φ*_*i*,*m*_^*h*^.

(24) $$\begin{array}{c} x_{m,i}^{c}=\frac{1}{\left(1+e^{-\sum_{i=1}^{J}\varphi_{im}}\right)}. \end{array}$$

Equation (24) is an expression of the principle of maximum fitness, the parameter *x*_*m*,*i*_^*c*^ is used to output the expected value of the sample corresponding to the connection point in the output network, the weighted value corresponding to the output connection point is represented by *φ*_*im*_, and the total number of layers in the output network is represented by *J*.

(25) $$\begin{array}{c} D\left(Z_{i}\right)=t-{optimal}_{i}\times \frac{1}{J}\overset{J}{\underset{i=1}{\sum }}\overset{q}{\underset{m=1}{\sum }}{\left(x_{m,i}^{c}-x_{m,i}\right)}^{2}. \end{array}$$

In equation (25), *D*() represents the calculation method of the mean square error, and the minimum principle is applied. In the network output, *q* is used to represent the total number of neurons, and *x*_*m*,*i*_ is the real parameter value of the sample, which is located at the output connection point in the network output. In this way, the PSO algorithm can be combined with the BP neural network model to better improve the sample accuracy and reduce the relative error.

The article "Construction of College English Teaching Environment Assessment Model Based on BP Neural Network and Multiple Intelligence Theory" was retracted in 2023. Reasons: signs of a paper mill; suspected computer-generated content; unreliable results or conclusions; lack of ethics approval or compliance.

## 4. Experiment on MultiAssessment Model of College Teaching in English Based on BPNN

### 4.1. Investigation of Multiple Evaluation Models

In order to reflect the scientific nature of the multiassessment model constructed in this paper, this study selected three English classes of the 2021 level of a university as the research objects. The English teaching model of this paper was promoted and implemented in these classes, which spanned a semester, and a questionnaire survey was conducted among the students who received the study after the end of the English test at the end of the semester. All 136 questionnaires issued were recovered, and the actual number of valid questionnaires was 128.  Table 2 shows the specific results of the questionnaires.

Table 2 shows that most students are very satisfied with and experience English teaching this semester. More than 68% of the students expressed their approval for the classroom evaluation methods of cooperative learning, self-assessment, and mutual assessment, and less than 8% of the students with poor experience. It can be seen that the teaching evaluation model proposed in this paper is welcomed by most students, and students have stronger interest and greater motivation to devote themselves to English learning.

At the same time, while investigating students' satisfaction with English teaching, this paper also collects the final English comprehensive scores of a total of 136 students in three classes. The specific results are shown in Table 3.

It can be seen from Table 3 that the English scores of the students in the three classes are all above the passing line of 60. At the same time, nearly 80% of the students score above 80, and nearly one-third of the students score above 90. This is undoubtedly a success for English teaching. This paper then compares the grades of this semester with the final grades of the previous semester when they did not receive multiassessment teaching. The comparison is shown in Figure 5.

Figure 5 shows that students' English final grades have improved significantly compared with the previous semester, and students with weaker English foundation have made particularly outstanding progress. Not only has the number of failing grades dropped from 11 last term to 0 but the number of students in the 60-70 and 70-80 grades has also dropped significantly, replaced by a significant breakthrough in the number of high grades above 80. This shows that the teaching evaluation model proposed in this paper can greatly improve the students' English performance, and the improvement effect is obvious in the actual application of English teaching.

The article "Construction of College English Teaching Environment Assessment Model Based on BP Neural Network and Multiple Intelligence Theory" was retracted in 2023. Reasons: signs of a paper mill; suspected computer-generated content; unreliable results or conclusions; lack of ethics approval or compliance.

### 4.2. Application of BPNN in Multivariate Evaluation Mode

In order to evaluate the feasibility of applying the BPNN technology to the multivariate evaluation model, this paper combines the three-layer architecture of the BPNN model with the multivariate evaluation model, and sets the input layer connection points as the expected value, actual value, and relative error. The rate is four, and the total number of connection points in the hidden layer is obtained from the above equation, and the total number of connection points in the output layer corresponds to the input layer, which is set to 4. Thus, the experimental model structure based on BPNN can be obtained, and the teaching evaluation index of the three classes investigated in this paper is applied to this structure. The experimental results obtained are shown in Table 4.

As can be seen from Table 4, the error rate of class A is 0.98%, that of class B is 0.62%, and that of class C is only 0.45%. It can be seen that the error of the multivariate evaluation system based on the BPNN is relatively small, the network structure fitting effect is good, and the training effect has reached the standard.

In addition, in order to show the advantages of the related models based on the BPNN algorithm compared with other traditional algorithms, this paper selects 370 sets of related data of the multivariate evaluation system. It is divided into two groups a and b for two control experiments, which are, respectively, applied to the BPNN algorithm and the traditional model algorithm. The specific error rate performance is shown in Figure 6:

Figure 6 shows that, according to the error conditions of the two control groups, the error rate interval of the traditional algorithm model is between 0.15% and 0.4%, and the error rate interval span is large, and the error rate is generally maintained above 0.25%. The overall error rate of the BPNN model is between 0.11% and 0.29% of the data segment. Obviously, compared with the traditional algorithm, the error rate generated by the BPNN model is much smaller. Accordingly, the accuracy of the algorithm will be higher.

### 4.3. PSO-BPNN Applied to Multivariate Evaluation Mode

In the above experiments on BPNN, although the error rate has been maintained at a considerable state, there is still room for improvement in the number and quality of selected samples. The experimental error does not meet the requirements of the teaching model system in this paper, and the experimental precision must be controlled in a higher range. In this case, this paper selects 10,000 pieces of data related to the indicators of the College English Teaching Multievaluation System as samples, 3,500 for random testing, and 6,500 for training samples. Figures 7 and 8 show the comparisons between the PSO-BPNN algorithm and the BPNN algorithm in terms of training time, number of iterations, error size, and accuracy, respectively. The test sample and the training sample are compared in order to achieve the effect of the objectivity and accuracy of the experimental data.

The article "Construction of College English Teaching Environment Assessment Model Based on BP Neural Network and Multiple Intelligence Theory" was retracted in 2023. Reasons: signs of a paper mill; suspected computer-generated content; unreliable results or conclusions; lack of ethics approval or compliance.

It can be seen from Figure 7 that in the training sample and the test sample, the error rate of the PSO-BP algorithm is always lower than that of the BPNN model under the comparison of the two algorithms with the same number of iterations. The error rate of the two in the initial stage is about 10^−1^, but with the increase of the number of iterations, the trend of the error rate is very different. In the training sample, when the number of iterations tends to 500, the error rate of PSO-BP is infinitely close to 10^−5^, while the BPNN model is 10^−3^. In the test sample, when the number of iterations tends to 300, the error rate of PSO-BP is also infinitely close to 10^−5^, but the BPNN model drops to 10^−2^.

Figure 8 shows the comparison of the relative error and average precision of the PSO-BP and BPNN models. For the same experimental object, the relative error of the BPNN is 0.47%, while the PSO-BPNN model controls the relative error to only 0.29%. Under the condition that the error is guaranteed to be extremely low, the PSO-BPNN model improves the average accuracy of the multivariate evaluation model system to 97.02%, while the BPNN model is only 86.79%. At the same time, the performance of the PSO-BPNN model in iteration time and training time is also significantly better than the BPNN algorithm. In terms of training time, the training time of the PSO-BP neural network model is only 198 seconds, which is much shorter than the 252 seconds of the BP neural network model. Experiments show that the PSO-BPNN algorithm has significant advantages in the study of multiple evaluation models in English teaching.

## 5. Conclusion

College English proficiency has always been an important indicator to measure students' learning ability and learning outcomes during college. However, in many colleges and universities, college teaching in English has always had many drawbacks that need to be solved urgently. This paper aims at the main contradiction that the current college English teaching is not diversified enough. This paper combines the theory of multiple intelligences with practical applications to construct a multiassessment model for college English. This mode is based on the BPNN model, which can improve the data accuracy very well. On this basis, combined with the further optimization of the PSO algorithm, this paper proposes an innovative PSO-BPNN algorithm. The relative error is only 0.29%, and the average accuracy is as high as 97.02%. It can well meet the high-precision requirements of the multivariate evaluation model, and it is a great help to improve the scientificity and accuracy of the multivariate evaluation model. In addition, the algorithm can also achieve the expected effect in reducing relative error but there is still some room for improvement. Therefore, in the follow-up work, this paper will focus on reducing the experimental error, and strive to minimize the error rate and keep it stable.

The article "Construction of College English Teaching Environment Assessment Model Based on BP Neural Network and Multiple Intelligence Theory" was retracted in 2023. Reasons: signs of a paper mill; suspected computer-generated content; unreliable results or conclusions; lack of ethics approval or compliance.

## Figures and Tables

**Figure 1:** Composition of multiple intelligences theory.

**Figure 2:** Multiple evaluation system of college teaching in English.

**Figure 3:** The structure of the BPNN.

**Figure 4:** Schematic diagram of PSO-BPNN.

**Figure 5:** Comparison of students' English scores.

**Figure 6:** Comparison of error rate between traditional model and BPNN algorithm model.

**Figure 7:** Comparison of the error curves of the two algorithms.

**Figure 8:** Test sample simulation results comparison.

**Table 1:** Proportion of students' comprehensive English scores.

Multiple evaluation index	Grading range(point)	Proportion(%)
Final exam grade	0-100	50%
Midterm assessment results	0-100	25%
Teacher evaluation score	0-50	12.5%
Classmates evaluation score	0-25	6.25%
Self-score	0-25	6.25%

**Table 2:** Satisfaction survey of English teaching mode.

Question	Good	Ordinary	Bad
Attitudes towards collaborative learning	88	30	10
Attitude towards test mode	92	25	11
Attitude of participating in mutual evaluation	89	32	7
Impact of assessment model on English learning	102	10	6

**Table 3:** Students' English test scores this semester.

English test scores	The number of student	Percentage
90-100	45	33.09%
80-90	62	45.59%
70-80	21	15.44%
60-70	8	5.88%
<60	0	0

**Table 4:** Teaching evaluation index prediction error for three classes.

Class name	Predictive value	Actual value	Error	Error rate (%)
A	211.8	209.5	2.3	0.98
B	223.8	222.4	1.4	0.62
C	267.4	266.2	1.2	0.45

## Data Availability

The dataset used to support the findings of this study are available from the corresponding author upon request.
